The article "Monitoring of Anesthesia by Bispectral Analysis of EEG Signals" was published in 2021. Journal: Comput Math Methods Med.

# Monitoring of Anesthesia by Bispectral Analysis of EEG Signals

**DOI:** 10.1155/2021/9961998

**Published:** 2021-09-20

**Authors:** Lamia Bouafif

**Affiliations:** National Institute of Biomedical Studies of Tunis-Image and Signal Processing Laboratory ENIT, University of Tunis Manar, Tunisia

## Abstract

**Background:**

In intensive care, monitoring the depth of anesthesia during surgical procedures is a key element in the success of the medical operation and postoperative recovery. However, despite the development of anesthesia thanks to technological and pharmacological advances, its side effects such as underdose or overdose of hypnotics remain a major problem. Observation and monitoring must combine clinical observations (loss of consciousness and reactivity) with tools for real-time measurement of changes in the depth of anesthesia. *Methodology*. In this work, we will develop a noninvasive method for calculating, monitoring, and controlling the depth of general anesthesia during surgery. The objective is to reduce the effects of pharmacological usage of hypnotics and to ensure better quality recovery. Thanks to the overall activity of sets of neurons in the brain, we have developed a BIS technique based on bispectral analysis of the electroencephalographic signal EEG. *Discussion*. By collecting the electrical voltages from the brain, we distinguish light sleep from deep sleep according to the values of the BIS indicator (ranging from 0 : sleep to 100 : wake) and also control it by acting on the dosage of propofol and sevoflurane. We showed that the BIS value must be maintained during the operation and the anesthesia at a value greater than 60.

**Conclusion:**

This study showed that the BIS technology led to an optimization of the anesthetic management, the adequacy of the hypnotic dosage, and a better postoperative recovery.

## 1. Introduction

Clinical monitoring is based on the analysis of nervous reactions to stimulation movements such as responsiveness to surgical incision and loss of verbal contact. The consequences of an unsuitable anesthesia are an increase in morbidity, overdosage. (hypotension and respiratory depression), or underdosage (memorization, movement, hypertension, and bronchospasm) [1].

This makes it essential to evaluate the depth of the anesthesia in order to optimize its adequacy to the intensity of the operative stimuli. Historically, the measurement of the depth of anesthesia began with the analysis of the relationship between nociceptive stimuli and the presence or absence of clinical signs such as loss of consciousness, movement, changes in respiratory rate, changes in eye response, and cardiovascular effects. It was in 1875 that an English doctor recorded for the first time the electrical potential of a brain.

In 1929, electroencephalography was invented by a German physician called Hans Berger, in order to study the electrical activity of the brain by measuring the electrical potential. This invention was recognized and completed by the physician Edger Adrian in 1934 [2].

In fact, the use of anesthesia depth monitoring emerged following a recommendation from the American Society of Anesthesiologists (ASA) in 2006, then a Cochrane Library meta-analysis in 2007 and a formal recommendation from SFAR experts in 2009. After 2000, two major studies of Liu's and Punjasawa Dwong's were carried out.

1. The first one includes 1380 patients from 11 outpatient surgery studies. It found a decrease in hypnotic's consumption of 19%
2. The second one includes 4056 patients from 20 studies. It found a decrease in propofol consumption of 1.30 mg/kg/h and a decrease in halogenated by 0.17 CAM equivalents [3]

Despite the existence of several BIS monitors, several of them suffer from problems such as low signal-to-noise ratio, artifacts, interference with EMG signals, and a medium precision of around 60% to 80%. In order to surmount these problems, we developed an embedded noninvasive BIS system for monitoring and control the depth of anesthesia during surgery. The first contribution is that we replaced the analog filtering, converters, and electrical circuits with programmable digital filters and embedded algorithms that are implemented in the Raspberry Pi4 electronic board. This avoids inaccuracies of the instrumental circuits and reduces artifact effects. The second contribution is that we succeeded to estimate from the simulation software the optimal dose of hypnotics to achieve a well-determined degree of sleep (for example: BIS = 30%), unlike other BIS monitors which adapt the anesthesia boluses with the evolution of BIC values.

### 1.1. Principle of Electroencephalography EEG

Electroencephalography is a recording of electrical activity in the brain. It represents the trace of temporal variation of electric potential collected on the cranial box for different points of the scalp. The EEG acquisition modality facilitates the visualization of the functioning of the cerebral process and the understanding of neurophysiological phenomena. The acquisition of the EEG signals is carried out from electrodes brought into contact with the scalp.

As EEG is a measure of brain electrical activity, its realization can occur during sleep or in other areas of activity. The received signal is very weak (some microvolts). It varies according to age, sex, the patient state, and alertness.

### 1.2. Electrical Activity

The brain is a building of a collection of nerve cells called neurons. They are very numerous, around tens of millions. They have the role of circulating nervous messages. Neurons have a long lifespan, and its electrical activity goes through two main phases:

1. Brain activity to neuron
2. Surface activity

### 1.3. Brain-to-Neuron Activity

The electrical activity of neurons depends on the polarization and depolarization of excitable cells. An action potential is a biphasic wave of a few milliseconds, which propagates towards all the nerve cells. It affects human activity such as perception, sleep, and memorization. The information value of the action potential is not transmitted by its amplitude but by its frequency. Therefore, with a depolarization above the threshold, the frequency of the action potential is the highest (Figure 1).

In Figure 1, neuron “ A ” represents the effect of two microelectrodes placed in the neuron. The first one injects current and the other records the membrane potential. The effect of this stimulation is summarized into 4 portions (B, C, D, and E). Portion B represents a result of a negative current, and the neuron is hyperpolarized.

No action potential is produced. Portion C represents a result of a positive current stimulation, depolarization of the neuronal membrane takes place but it is not sufficient to generate an action potential. For portion D, the injected current depolarizes the membrane to a value greater than the threshold. An action potential is generated. Finally, the discharge frequency of the action potentials will be high with the level of depolarization, proportional to the quantity of current injected; this is the case of portion E.

### 1.4. Surface Activity

Between two neurons, the interface zone is a surface with a porous membrane which allows the exchange of sodium, chlorine, potassium, and ions. Subsequently, the appearance of an ionic current is observed which propagates towards various cells with a precise frequency. The efficiency of information transfer from one region to another brain level depends mainly on the activity level of the cortex. As an action potential propagates along an axon, Na+ ions enter the cell at the active site through voltage-gated Na+ channels. On either side of this depolarization front, a flow of K+ ions emerges via channels open at rest or with delayed opening. As illustrated in Figure 2, this active axonal portion can be assimilated to a current quadruple (two inverted dipoles) [2].

According to the following Figure 3, the polarization of the EEG waves in the surface depends on the position of the synapse in active mode. In fact, the deviation of the potential upwards indicates a negative potential, and conversely, the deviation in the opposite direction indicates a positive potential.

Any EEG electrical signal is characterized by its frequency and its amplitude: the frequencies are between 0.5 to 40 Hz and the amplitude varies from 5 to 250 microvolts.

In general, amplitudes and frequencies are calculated over a period of 125 ms to 20 s.

For example, Figure 4 shows an EEG signal recorded by electrodes placed on the scalp surface. We obtained a weak electric field produced mainly by synaptic potentials which can be classified as synchronized waves (c) or irregular: not synchronized (b).

## 2. Materials and Methods

### 2.1. Description of the Vigilance and Sleep States

Since the development of exploiting electrical activity, the experimental approach to sleep has become scientific. Billiard [5] was the first to identify the state of alertness and sleep during the night. Each state of vigilance corresponds to a specific potential and the use of three parameters (waking state, light and slow sleep state, and slow and deep sleep state). The signal processing of the EEG signal identified five cerebral rhythms: Delta, Theta, Alpha, Beta, and Gamma. These rhythms are classified according to their frequency band and their amplitude according to Table 1.

The temporal waveforms of brain waves are illustrated in Figure 5.

#### 2.1.1. Standby State

It is the stage which characterizes the discontinuous emission of alpha wave. We therefore observe a reduction in amplitude which results in the alpha wave flattening.

There are two standby states:

1. The first is active awakening characterized by the appearance of low amplitudes between 5 and 20 microvolts with a rapid frequency. We are talking about beta wave
2. However, the second state is calm awakening which corresponds to the alpha wave

#### 2.1.2. Slow and Light Sleep State (Figure 6)

It is characterized by a slowing of brain waves with an increase in amplitude, and it breaks down into four stages of increasing depth:

- *Stage 1*. Is a stage between wakefulness and sleep corresponding to theta wave: 10% of sleep in young adults
- *Stage 2*. Is a confirmed sleep exhibiting the characteristics of a slow theta wave by breaking down into two types of waves. The first is a sleep spindle wave at a fast (12 to 16 Hz) and short-term (1 to 2 s) frequency. The second is characterized by the slow wave and appears in a transient and cyclical way
- *Stage 3 and 4*. The two stages are deep sleep. It presents the characteristic of slow wave delta with higher amplitude than 75 microvolts and a frequency range between 0.5 and 4 Hz

#### 2.1.3. Slow and Deep Sleep State (Figure 7)

An essential stage in children because it is the period of secretion of growth hormone which activates all the synthesis processes from the early morning, in particular the protein. The paradoxical slow sleep presents an active center of the hypnogram. It is with the paradoxical sleep that one obtains the expression of the regenerative functions of dream and sleep.

#### 2.1.4. REM Sleep State (Figure 8)

This stage of sleep is slow and paradoxical (also called PMO stage, eye movement phase, or REM*).* This state is shorter with an intensive brain activity. This period is accompanied by rapid eye movement caused by brain waves, which is related to dreams. This hard sleep is between 15 to 20 minutes. It is characterized by low amplitude and rapid pace. It appears for a movement ordered but not realized and louse thought lively, strange, and illogical [8].

### 2.2. Registration Procedure by Electrodes

For EEG signal acquisition, the sensors are electrodes which record the variations in electrical potential which are a few millimeters in radius. The electrodes are inserted in an elastic cap. The bonnet that is placed on the head of a patient is decomposed of a tissue and electrodes. The electrodes are of the “Gray-Walter” type which consists of a silver rod covered with a tissue plug inhibited by a saline solution. They are fixed in a stabilizing support which allows them to stand upright on the scalp. They are held by a small hook which is a net made in the crisscrossed rubber strap that is fixed on the subject's head in order to keep the electrodes in suitable places. As illustrated in Figure 9, each letter indicated on the electrodes a specified region. Even numbers indicate the right side and the odd numbers indicate the left dimension.

#### 2.2.1. Rhythmic Activity

The form and intensity of EEG electrical activity depend on the position of the recording electrodes and on brain activity (Figure 10). They depend on the location of the electrodes, their impedances, and the state of sleep. Electroencephalography (EEG) is used to record the rhythmic activities of the cerebral cortex, classified into five waves: Delta, Theta, Alpha, Beta, and Gamma [9].

### 2.3. The BIS Procedure

The study of the energy spectrum of cortical signals shows the existence of frequency bands that are related to behavioral observations. The frequency waves are divided as follows [10]:

1. Delta band (0 to 4 Hz)
2. Theta band (4 to 8 Hz)
3. Alpha band (8 to 12 Hz)
4. Beta band (12 to 25 Hz)
5. Gamma band (>30 Hz)

Power spectral analysis gives information on amplitude and frequency but does not take into account the phase between the components of different frequencies. The first-order statistics lose all phase information. In order to retrieve the statistical information, we introduce the bispectral analysis [11].

### 2.4. Bispectral Analysis

#### 2.4.1. Quadratic Phase Coupling (QPC)

To be able to quantify the quadratic phase coupling between pairs of frequencies, it is necessary to calculate from bispectrum. The interaction of two wave trains of frequencies *f*1 and *f*2 can generate two interaction waves of frequencies (*f*_1_ + *f*_2_) and (*f*_1_ − *f*_2_).

The frequency components can therefore interact and produce other mixed frequency components whose wave numbers and frequencies are formed from the sum or the difference of these primary components. The frequencies *f*_1_, *f*_2_, and *f*_3_ can be related by a quadratic nonlinear interaction if the following equation is satisfied [12]:

(1) $$\begin{array}{c} f_{1}\pm f_{2}\pm f_{3}=0. \end{array}$$

In general, if we have a signal which is composed of three sinusoids with frequencies and phases (*ω*1, *ϕ*1), (*ω*2, *ϕ*2), and (*ω*3, *ϕ*3), the sinusoids 1 and 2 are said to be quadratically coupled in phase (QPC) if and only if [13]:

(2) $$\begin{array}{c} \omega 1\pm \omega 2\pm \omega 3=0, \end{array}$$

(3) $$\begin{array}{c} \varphi 1\pm \varphi 2\pm \varphi 3=0 \end{array}$$

### 2.5. Bispectrum and Bicoherence

The bispectrum is a complex quantity that measures nonlinear interactions in a process that generates a signal and the correlation between the phases of a signal at different Fourier frequencies. So the analysis bispectral is defined as a FFT-2D, and bispectrum is the Fourier transform of the sequence of third order cumulate of a random process.

Despite its capacity for calculation, the bispectrum remains complex to understand it. It is for this reason one calls upon the bicoherence [11]. This index varies between 0% and 100%.

#### 2.5.1. Calculation of the Bispectrum

To compute the bispectrum, EEG signals are first divided into a series of epochs. Then, Fourier transform *X*_*j*_(*f*) of each epoch is computed. The bispectrum *B*(*f*_1_, *f*_2_) is calculated from the following equations:

(4) $$\begin{array}{c} \text{T}{\text{P}}_{j}\left(f_{1},f_{2}\right)=X_{j}\left(f_{1}\right).X_{j}\left(f_{2}\right).X_{j}^{*}\left(f_{1}+f_{2}\right), \end{array}$$

(5) $$\begin{array}{c} \;B\left(f_{1},f_{2}\right)=\left|\underset{j}{\sum }\text{T}\text{P}j\left(f1,f2\right)\right|, \end{array}$$

where TP_*j*_ is the spectral triple product. *X*(*f*_1_), *X*(*f*_2_), and *X*(*f*_1_ + *f*_2_) are complex values calculated from Fourier transform.

*X*∗(*f*) is the conjugate of *X*(*f*).

For real processes, there are 12 areas of symmetry in the bispectrum [14]. The bicoherence BIC is defined as the degree of standardized BIS (between 0% and 100%). The normalized value of the bispectrum is called bicoherence BIC(*f*_1_, *f*_2_). It is calculated from the following equation [15]:

(6) $$\begin{array}{c} \text{ BIC}\left(f_{1},f_{2}\right)=\frac{B\left(f_{1},f_{2}\right)}{\sum_{j}\left|\text{TP}j\left(f_{1},f_{2}\right)\right|}.100, \end{array}$$

The numerator is different from the denominator because:

(7) $$\begin{array}{c} \left|\sum \text{T}{\text{P}}_{j}\right|\leq \sum \left|\text{TP}j\right|. \end{array}$$

This expression can be expressed in function of the power spectral density *P*(*f*) as:

(8) $$\begin{array}{c} \text{ BIC}\left(f_{1},f_{2}\right)=\frac{B\left(f_{1},f_{2}\right)}{\sum_{j}\sqrt{Pj\left(f_{1}\right).Pj\left(f_{2}\right).Pj\left(f_{1}+f_{2}\right)}}.100. \end{array}$$

The last formula can be deduced as:

(9) $$\begin{array}{c} {\left|\text{T}{\text{P}}_{j}\left(f_{1},f_{2}\right)\right|}^{2}={\left|X_{j}\left(f_{1}\right)\right|}^{2}.{\left.X_{j}\left(f_{2}\right)\right|}^{2}.{\left|X_{j}^{*}\left(f_{1}+f_{2}\right)\right|}^{2}=P_{j}\left(f_{1}\right).P_{j}\left(f_{2}\right).P_{j}\left(f_{1}+f_{2}\right). \end{array}$$

Then

(10) $$\begin{array}{c} \;\left|{\text{TP}}_{j}\left(f_{1},f_{2}\right)\right|=\sqrt{P_{1}\left(f_{1}\right).P_{j}\left(f_{2}\right).Pj\left(f_{1}+f_{2}\right)}. \end{array}$$

With the power spectral density *P*_*j*_(*f*) = |*X*_*j*_(*f*)|^2^.

## 3. Results and Discussion

Figure 11 illustrates the principle of the EEG segmentation and wave's discrimination. We start by reading the data from the EEG recordings which are saved in a called “file_name.edf”.

Then, the EEG signal is into frames of 512 points with a sampling frequency of 500 Hz. We thus obtain the cerebral rhythms (Alpha, Beta, Theta, Delta, and Gamma). Finally, we apply the fast Fourier transform (FFT) in order to separate and to identify the 5 waves: Delta (0-4 Hz), Theta (4 to 8 Hz), Alpha (8-12 Hz), Beta (12 to 30 Hz), and Gamma (>30 Hz).

### 3.1. Simulation

The following Figures 12–16 represent the results of the spectral analysis of the EEG signals, called the brain waves. Every one of these five signals represents a specific state of the patient.

Figure 17 shows the spectral density of the EEG signal. The beta wave portion is characterized by a peak, observed at 30 Hz. The beta brain wave appears in a patient with open eyes and for a frequency of 12 to 30 Hz. The obtained results show that from calculation of the spectral density of the signal, it is possible to identify the patient case where it is not always sufficient.

### 3.2. Database and Experiment Protocols

In section, we will study two different signals in order to detect quadratic phase coupling:

- The first signal processed is an EEG examination result for a healthy patient (male, 25 years old: not affected by neurological diseases such as epilepsy), calm with open eyes
- The second signal processed from a patient (26-year-old woman) under anesthesia (with 2.6% sevoflurane)

The protocol for the measurements is as follows:

- EEG signals are collected from electrodes placed at defined locations on the scalp. The placement of the electrodes is defined according to Figure 9
- We used the 10-20 system because it identifies the same relative position on the scalp regardless of head size. It is based on meridians crossing the scalp into landmarks such as nasion, inion, left, and right auditory tragus

The “10-20” refers to the fact that actual distances between adjacent electrodes are either 10% or 20% of the total front-back or right-left distance of the skull (Figure 9). Each electrode placement site has a letter to identify the lobe, or area of the brain: the standard positions and areas are classified as illustrated in Figure 18: prefrontal (Fp), frontal (F), temporal (T), parietal (P), occipital (O), and central (C). There are also (*Z*) sites for electrodes placed on the midline sagittal plane of the skull, (Fz, Cz, Pz, and Oz) which are present mostly for reference-measurement points. Even-numbered electrodes refer to electrode placement on the right side of the head, whereas odd number electrodes refer to the left side.

- Electrode-gels are used. They act as a malleable extension of the electrode, so that the movement of the cables is less likely to produce artifacts. The gel maximizes skin contact and allows for a low-resistance recording through the skin
- To eliminate the offsets, the voltage is defined as the potential difference between 2 electrodes, grouped by 2. Among the 20 sensors, four electrodes were selected: Fp1-Fp2 and T3-T4

This choice is justified by the ease of access to contact points and the symmetry with respect to the middle head.

The impedance of each electrode is in the order of 1000 ohms.

- For signal amplification, we used differential amplifiers. They magnify the difference between two channels or electrodes. The advantage is that, an unwanted signal which is common to the two inputs will be subtracted
- Many signals present on the scalp, include power line interference at 50 Hz and the electromyogram EMG, which may extend above 100 Hz. To prevent aliasing distortion of the EEG signal, we adopt a sample rate above 250 Hz (Fs = 500 Hz in our case). The filtering is based on a second-order band pass I.I.R digital filter [1 Hz; 75 Hz] to respond to the Nyquist frequency Fn = Fs/2 (Fn = 250 Hz) and to restore alpha, beta waves, gamma, delta waves, and also to eliminate artifacts and network harmonics (Figure 19).

The filter bank is based on a decomposition into five IIR bandpass filters (BPF) related to the EEG waves (delta, theta, alpha, beta, and gamma) followed by a downloading step by a factor 2. The five output signals are applied to a preprocessing step constituted by a deconvolution of artifacts/EEG and EMG/EEG by using the cepstral method. Finally, we can restore the enhanced EEG signals by low-pass filters (LPF).

### 3.3. Algorithm of the BIS Application on the EEG Signal

After the first step of reading data from EEG, the output signals are saved as “∗.edf” file. Then, the EEG file is segmented into 512 points per frame with a sampling frequency of 500 Hz. The estimation of HOS is computed by the bispectrum analysis in order to detect the phase of quadratic coupling between the various components of EEG signal. Finally, the normalization of the bicoherence of the bispectrum result was calculated, between 0 and 100%.

This algorithm is similar to PLE (phase lag entropy) that uses four-channel EEG to measure the temporal pattern diversity in the phase relationship of frequency brain signals [16, 17].

Figure 20 illustrates the principle of the BIC algorithm. We begin with the analysis of the EEG signal of the patient with open eyes by reading the signal with a sampling frequency Fs = 500 Hz and a frame length = 512 samples. Note that when we calculated the spectral power of an awake subject, it is found a peak of 30 Hz corresponding to the beta brain rhythms. Our aim in this section is to count the quadratic phase coupling QPC. This function detects the quadratically coupled harmonics in phase using the TOR method (third-order recursion) and calculates the bispectrum value of the coupled components. The following figure shows the EEG signal bispectrum of an awake breast subject.

### 3.4. Simulation Results

The parametric estimation of the bispectrum shows the presence of weak phase coupling (blue outline in Figure 21) between the different components of the EEG signal of the awake patient with a maximum of bispectrum located at the point B (0.0976, 0.0117). The bispectrum result should be normalized across the bicoherence or bispectrum normalized through the BIC equation: BIC = 92.2%.

Subsequently, we are interested in analyzing the EEG signal of the patient under anesthesia (2.6% sevoflurane [18]) by reading the signal which is normalized at the same conditions. Note also when we calculated the spectral power of subjects under anesthesia, we found a peak of 2 Hz corresponds to the cerebral rhythm delta. The following Figure 21 shows the bispectrum of the EEG signal of a patient under anesthesia (2.6% sevoflurane).

The parametric estimation of the bispectrum shows the presence of a strong phase coupling (presence of red outline in Figure 22) between the different components of the EEG signal of the awake patient with maximum of bispectrum, located at B (0.49609, 0.24609), and the presence of other value is given by B (0.1312, 0.1351), (0.2385, 0.1487), B (0.2502, 02460). The bicoherence or normalized bispectrum is BIC = 3.1%. We notice in last Figures 21 and 22 the absence of quadratic coupling for the awake breast patient with a normalized value of BIC = 92.2% (Figure 21) and a strong presence of coupling in the patient under anesthesia of a value of BIC = 3.1% (Figure 22).

Table 2 summarizes the obtained values and results.

The identification ratio of our tests is summarized in the following Table 3.

We can interpret that going towards the value 100% the marked subject awake with an absence of phase coupling and going towards 0% the subject marked under anesthesia with a strong presence of coupling. The absence of coupling computed by the bispectrum signifies patient awareness, and the strong presence of coupling signifies the vigilance of the patient. Finally, with our strategy, we obtained an accuracy of 92% which is very promising and interesting, one compared with other industrial BIS or entropy monitors.

### 3.5. Comparison with Other Studies

In Table 4, we compared our results with three similar bibliographic studies using as judgment parameters, the sedation-awakening period, the percentage of morphine or sevoflurane, the BIC error, and the number of doses taken during anesthesia. We notice that we obtained similar results to Zhao's study with a decrease in error and consciousness recovery time.

## 4. Conclusion

The study of EEG signals is very complex because it requires the knowledge of biological brain signals and the technologies relating to its components. The aim of this study is to develop a noninvasive method for computing and monitoring in real time the degree of general anesthesia by applying the bispectral analysis of the EEG signal. We developed a methodology of EEG signal segmentation and bispectral analysis in order to extract the five brain waves.

We demonstrated that every wave corresponds to a specific state of the patient. In order to identify the patient state, during and after anesthesia, we computed the synchronization between the components of the spectrum by using the quadratic phase coupling (QPC) strategy. The obtained values of the bispectrum and bicoherence index allowed us to classify and then to recognize the patient state and the anesthesia evolution. These results are very interesting because they can assist medical staff to better control and monitoring the anesthesia during surgery operations, reduce the use of hypnotics, and contribute to a better postoperative recovery.

## Figures and Tables

**Figure 1:** Principle of the action potential [3].

**Figure 2:** Action potential propagation diagram [2].

**Figure 3:** The principle of EEG registration [3].

**Figure 4:** EEG signals related to synaptic activity [4].

**Figure 5:** Illustration of brain waves [6].

**Figure 6:** EEG waveforms of the slow and light sleep stage [7]. (1): EEG signal, (2): left eye, (3) right eye, (4) EMG.

**Figure 7:** Profile of the GET step of slow and deep sleep [7].

**Figure 8:** Profile GET step of REM sleep [7].

**Figure 9:** Localization of EEG electrodes [7]. F: frontal; Fp: polar front; A: earlobe; C: central; O: occipital; T: temporal; Z: central axis; P: parietal.

**Figure 10:** EEG measuring system during eye movements [6] (closed, opened).

**Figure 11:** Wave extraction algorithm.

**Figure 12:** The delta wave: deep sleep.

**Figure 13:** The theta wave: light sleep.

**Figure 14:** Alpha wave: brain sleeping

**Figure 15:** Beta wave: first activity/eye's opening.

**Figure 16:** The gamma wave: information processing.

**Figure 17:** Spectral density of an extract of the EEG signal.

**Figure 18:** Electrodes positions.

**Figure 19:** Filterbank decomposition of EEG signals.

**Figure 20:** BIS and BIC algorithm of an EEG signal.

**Figure 21:** Bispectrum with open eyes.

**Figure 22:** Bispectrum of a patient under anesthesia (2.6% sevoflurane).

**Table 1:** Characteristics of brain waves.

Wave	Physio/psycho	Frequency (Hz)	Amplitude (*μ*V)
Delta	-Deep sleep Eye movement: abnormal	0-4	300
Theta	-Light sleep -Eyes closed	4-8	50-100
Alpha	-Mental calm Receptivity, relaxation -Eyes closed	8-12	30-50
Beta	-Paradoxical sleep -Rational thinking -Eyes open -Vigilance	12-30	10
Gamma	-Simultaneous information from different sectors -Problem resolution	>30	—

**Table 2:** Comparison table between the value of BIS and the value found.

Patient state	Theoretical BIS value in %	Real value in %
Patient under awake state	100	92.2
Patient under anesthesia	0	3.1

**Table 3:** Identification rate table between the two patient cases.

Patient condition	Awake	Under anesthesia
Identification ratio (%)	90.4	96.6

**Table 4:** Comparison with similar BIS studies.

Reference study	Average propofol dose (mg/kg/hour)	Time to consciousness (minutes)	Average number of boluses	Mean error
Inaba et al. [19]	5.3	5.7	2.3	0.2
Weatherburn et al. [20]	18.4	14.6	—	0.67
Zhao et al. [21]	0.95	15	—	0.09
Lamia (our study)	2.6	3.2	1	0.03

## Data Availability

Data used in this work are from references and free databases mentioned in the text

## Abbreviations

BIS: Bispectral index
BIC: Bicoherence index
EEG: Electroencephalography
QPC: Quadratic phase coupling
SFAR: French Society of Anesthesia and Reanimation
ASA: American Society of Anesthesiologists.
